The article "Genome-wide association mapping for high temperature tolerance in wheat through 90k SNP array using physiological and yield traits" was retracted in 2023. Reasons: a conflict of interest; concerns about the peer review; concerns about the authorship.

# Genome-wide association mapping for high temperature tolerance in wheat through 90k SNP array using physiological and yield traits

**DOI:** 10.1371/journal.pone.0262569

**Published:** 2022-01-14

**Authors:** Hafiz Ghulam Muhu-Din Ahmed, Muhammad Naeem, Yawen Zeng, Muhammad Abdul Rehman Rashid, Aziz Ullah, Amjad Saeed, Abdul Qadeer

**Affiliations:** 1 Department of Plant Breeding and Genetics, Faculty of Agriculture and Environment, The Islamia University of Bahawalpur, Pakistan; 2 Biotechnology and Germplasm Resources Institute, Yunnan Academy of Agricultural Sciences, Kunming, China; 3 Department of Bioinformatics and Biotechnology, Government College University Faisalabad, Pakistan; 4 Department of Plant Breeding and Genetics, University of Sargodha, Sargodha, Pakistan; 5 Department of Forestry Range and Wildlife Management, Faculty of Agriculture and Environment, The Islamia University of Bahawalpur, Bahawalpur, Pakistan; 6 Soil Fertility and Plant Nutrition Laboratory, Institute of Soil and Environmental Sciences, University of Agriculture Faisalabad, Faisalabad, Pakistan; Sivas Bilim ve Teknoloji Universitesi, TURKEY

## Abstract

Dissecting the genetic basis of physiological and yield traits against tolerance to heat stress is an essential in wheat breeding programs to boost up the wheat yield for sustainable food security. Herein, a genome-wide association study (GWAS) was performed to reveal the genetic basis of heat tolerance using high-density Illumina 90K Infinium SNPs array through physiological and yield indices. These indices were phenotyped on a diverse panel of foreign and domestic genotypes of Pakistan, grown in normal and heat-stressed environments. Based on STRUCTURE analysis, the studied germplasm clustered into four sub-population. Highly significant variations with a range of moderate (58.3%) to high (77.8%) heritability was observed under both conditions. Strong positive correlation existed among physiological and yield related attributes. A total of 320 significant (-log10 P ≥ 3) marker-trait associations (MTAs) were identified for the observed characters. Out of them 169 and 151 MTAs were recorded in normal and heat stress environments, respectively. Among the MTA loci, three (*RAC875_c103017_302*, *Tdurum_contig42087_1199*, and *Tdurum_contig46877_488* on chromosomes 4B, 6B, and 7B respectively), two (*BobWhite_c836_422* and *BS00010616_51*) and three (*Kukri_rep_c87210_361*, *D_GA8KES401BNLTU_253* and *Tdurum_contig1015_131*) on chromosomes 5A, 1B, and 3D at the positions 243.59cM, 77.82cM and 292.51cM) showed pleiotropic effects in studied traits under normal, heat-stressed and both conditions respectively. The present study not only authenticated the numerous previously reported MTAs for examined attributes but also revealed novel MTAs under heat-stressed conditions. Identified SNPs will be beneficial in determining the novel genes in wheat to develop the heat tolerant and best yielded genotypes to fulfill the wheat requirement for the growing population.

The article "Genome-wide association mapping for high temperature tolerance in wheat through 90k SNP array using physiological and yield traits" was retracted in 2023. Reasons: a conflict of interest; concerns about the peer review; concerns about the authorship.

## Introduction

Wheat is one of the staple crop in the world, high and stable yield in this crop is an essential goal for growing wheat. Wheat has an optimum day-time growing temperature due to cool season crop during reproductive development of 15°C and for each degree Celsius more than optimal temperature a yield decrease of 3–4% were recorded [1]. However, the global average temperature is recorded, would increase at a rate of 0.18°C every ten years [2]. Climate change is causing not only an increase in global average temperatures, but also the more frequent occurrence of extreme weather events [3]. The averaged Earth’s surface temperature risen about 0.85°C from 1880 to 2012 and is forecast to continuously increasing [4]. To develop the heat tolerant wheat genotype, it is necessary to explore desired alleles to use in breeding programs.

The actual grain yield of wheat crop does not match to its potential due to several restricting factors, one of which is heat stress [5]. Several scientists observed a 50–90% reduction in wheat yield under heat stressed conditions as compared to its genetic potential in different areas of the world [6–8]. The demand for wheat continuously increasing with the constant growth of the human population and is expected to rise up to 40% till 2030. So, increased grain yield is an imperative need to establish food security [9–11]. Wheat cultivation ranks first between another cereal grain crops because it has more nutritional values and maximum uses. Rapid population growth and a healthier lifestyle have created new responsibilities for wheat scientists to develop wheat varieties having high yield, best quality and resistance to a-biotic and biotic stresses to ful fill the wheat requirement [12, 13].

Heat tolerance is a complex and polygenically controlled character that is influenced by numerous genes with a minor impact on the morphology of plant. Hence, the selection of tolerance to heat stress in field conditions is very difficult due to its genetically complex, meteorological variations and the effect of genotypes-environment interactions. In such a manner, the identification of quantitative trait loci (QTLs) and molecular marker linked with heat stress tolerance is essential to improve breeding efficacy through marker-assisted selection (MAS) [5, 7]. Heat stress is a complex mechanism due to it relies on numerous factors, such as the cultivated species, the intensity of the heat stress, the duration of the heat stress and the stages of plant growth [14]. To create high temperature tolerant wheat genotypes, it is very important to know the plant mechanism and performance under heat stress environments. Even though breeding development for the advancement in wheat has been accomplished for non-stressed conditions, but less achivements have also been obtained for heat stressed environments [10, 15]. Methods to reducing this gap comprise advancing genetics for heat stressed conditions and the ensuing introgression of gene for certain traits associated with locally cultivated wheat genotypes. The tasks in applying such methods in breeding programs are knowing the characteristics required in an efficient and cost effective technique against heat stress conditions [1, 6, 16].

The article "Genome-wide association mapping for high temperature tolerance in wheat through 90k SNP array using physiological and yield traits" was retracted in 2023. Reasons: a conflict of interest; concerns about the peer review; concerns about the authorship.

Producing of maximum yielded and heat stress tolerant genotype is difficult by numerous complications because yield and heat stress tolerance associated genes are polygenic and complex in nature. Several procedures were practiced for choosing the spring wheat genotypes for heat stress environments. Rehman et al [17] suggested cell membrane thermo-stability trait (CMT) in wheat crop to use as selection criteria against heat stress resistance. Several scientists [18] also reported that this trait in wheat is a best criteria for choosing the heat stress tolerant genotypes. ElBasyoni et al [13] conducted a study in normal and heat stressed environments and selected heat stress-tolerant varieties, which had optimum CMT in wheat. Screening of wheat genotypes based on the heat stress-related characters is informal, easy, quick and low-cost [4, 19].

The effect of stimulation to heat stress was studied with maximum crop canopy temperature. Canopy temperature (CT) at vegitative and reproductive stage is main character that is used by a breeder to select best wheat lines against tolerance to heat as well as drought stress [20]. Grain yield show positive correlation with canopy temperature, which showed that canopy temperature always has a role in grain yield of wheat [21]. Heat stress during anthesis damages the reproductive organs associated with spike fertility. High temperatures hinder the micro-sporogenesis and micro-gametogenesis which induce spore abortion subsequently reduction in grain formation [22, 23]. It also inhibits starch accumulation into grains due to granule bound starch, soluble starch and sucrose synthase enzymes activity during grain filling that consequently leads to reduction in grain size, weight and ultimately grain yield. Grain filling duration and grain filling rate determines grain development. Longer grain filling duration facilitates the longer time to capture available resources and improve the grain weight. Days to heading (DH) is most important to determine life of plant and days taken for anthesis [24, 25].

The article "Genome-wide association mapping for high temperature tolerance in wheat through 90k SNP array using physiological and yield traits" was retracted in 2023. Reasons: a conflict of interest; concerns about the peer review; concerns about the authorship.

Numerous attempts were made using the conventional breeding strategies to improve wheat yield in heat stressed conditions, but these approaches have only contributed to an increase of more than only 1% in annual production [12, 14]. In coming days, the wheat breeding scheme will rely on findings the genetics and molecular potential against tolerance to heat stress through QTLs, GWAS and next generation sequencing (NGS). Therefore, identifying stable QTL / alleles for better performance in different environments is essential to tackle climate change [26]. GWAS with genotypically and phenotypically obtained data from associations panel have proven to be a vigorous technique for perceiving QTL associated with specific trait [27]. Enable the use of various sets of genetic material and make wider genomics regions / allele frequencies available with more resolutions, without any biparental population mapping [28]. GWAS discovers the genetic basis of desired traits and their associated genes. It is an important practice to have good outcomes due to the more genetic diversity (GD) contained and the promising recombinant allele within the appropriate panel [29]. It is also valuable to detect genomic regions linked to heat stress tolerance and desired attributes in various associations mapping panel.

In this study, a miscellaneous panel of wheat genotypes was genotyped with 90K SNPs array as well as phenotyped in non-stressed and heat stressed environments during 2 crop seasons in 2018–19 and 2019–20. This study delivers valued evidence about the genetics of tolerance to heat stress in wheat. Novel SNPs were observed to be related with key heat stress tolerant attributes. The significantly associated SNPs with physiological and yield indices would be useful to identify and mapping the candidate genes for heat stress tolerance in wheat.

## Materials and methods

Total 96 Pakistani and foreign (USA, Australia, Mexico and India) wheat genotypes were preserved at the Department of Plant Breeding and Genetics, University of Agriculture Faisalabad PBG-UAF that were used in this experiment. Complete data about the accessions code, their origin, the names and the pedigrees are mentioned in S1 Table in S1 File. Genotypes was seeded into two different sets of environmental conditions in triplicate with a randomized complete block design over two consecutive growing seasons 2018–19 and 2019–20. One set of genotypes sown in the tunnel and other set of genotypes was sown in the field under normal environment. Heat stress was applied to wheat plants at the anthesis stage by covering the tunnel using the plastic sheet. The temperature was observed daily on both internal and external sides of the tunnel and maintained at > 40°C internal side of the tunnel. Each genotype was seeded in an experimental unit having three replications while maintaining the P × P distance of 6 inches and the R × R distance of 12 inches. Only two seed of respective accessions have been planted / hole and maintained vigor seedlings by thinning at the time of two-leaf stage. All other agronomic applications like fertilizer applications, hoeing, weeding, etc., were used consistently to decrease experimental errors in studied environments. Data were observed from 10 plants of every replication for flag leaf area (FLA), cell membrane thermo-stability (CMT), canopy temperature at vegetative stage (CTV), canopy temperature at grain filling stage (CTG), day to headings (DH), day to maturity (DM), 1000-grain weight (TGW) and grain yield per plant in examined conditions. Length and width of flag leaf were calculated in cm^2^ in this study. Formula used for the calculation of flag leaf area described by Muller [30] as under.

The article "Genome-wide association mapping for high temperature tolerance in wheat through 90k SNP array using physiological and yield traits" was retracted in 2023. Reasons: a conflict of interest; concerns about the peer review; concerns about the authorship.

Flag leaf area = length of flag leaf × width of flag leaf × 0.74. Cell membrane thermo-stability (CMT) was measured by using the previously described procedure [31]. Two fully expanded leaves were taken from tagged wheat plants. Each leaf was cut into two pieces to consider as normal and as heat-treated. Halved leaves were subjected into two test tubes having 10 ml of distilled water for 18h at 10°C. After washing the leaves, 15 ml distilled water was added. Then, all the test tubes were put in water bath while the one half of each test tube was kept at 25°C and the other half at 45°C for 1 hour. Both normal and heated leaves were further kept for 18h at 10°C to maintain the contents. Conductivity data were scored at 25°C with an electrical conductivity (EC) meter for control (C1) and heated (T1) tubes. The leaves were again subjected to heat for 1h. Another conductivity data of the aqueous phase (T2 and C2) was observed at 25°C after cooling the leaves. Cell membrane thermo-stability (CMT) was also expressed as percent relative injury (RI%) [31].

$$\text{Cell}\;\text{membrane}\;\text{thermo}-\mathrm{stability},\;CMT\;\left(\%\right):\;\left[1-\;\left(T_{1}/T_{2}\right)\right]\times 100$$

$$Relative\;Injury\;\left(RI\right)\;\%\;=\;100-[\left[1-\left(T_{1}/T_{2}\right)\right]/[1-\left(C_{1}/C_{2}\right)]\times 100].$$

Where, C and T represent the electrical conductivity of normal and heated sample while the subscript 1 and 2 indicate electrical conductivity readings before and after autoclaved, respectively.

The article "Genome-wide association mapping for high temperature tolerance in wheat through 90k SNP array using physiological and yield traits" was retracted in 2023. Reasons: a conflict of interest; concerns about the peer review; concerns about the authorship.

Days to heading (DH) was counted from the date of sowing up to the date when it has above 50% plant with the complete heading. At booting stage of the crop, a hand-held digital Infrared thermometer LT300 is used to calculate canopy temperature at vegetative stage (CTV) in centigrade. The distance from the canopy was kept 50cm and the slope was 45°, taking care that laser light should only focus on the canopy and data was recorded on a sunny day from 10:00 a.m. to 2:00 p.m. Data were recorded for canopy temperature at grain filling stage (CTG) at mid grain filling stage with the help of infrared thermometer with the same procedure and precautions. From selected plants, days taken to maturity (DM) were examined as the duration from sowing to maturity dates when plants were physiologically mature. Ten plants were randomly selected from all replications of each entry and bulked separately. TGW were taken from bulk seeds and were weighted by using and electric balance (Compax- Cx-600) to record TGW. Threshing of all spikes from the selected plants than with the use of electric balance, (Compax- Cx-600) weighted. Mean data of grain yield/plant (GYP) was calculated from replications

### Statistical analysis

The noted data were applied for the combined analysis of variance (ANOVA) through the GenStat ® Ver.17 [32] for examined traits observed in normal and heat stressed conditions. “The broad sense heritability for each trait was calculated using the following equation [5, 29, 33]

$$H^{2}=\sigma_{g}^{2}/(\sigma_{g}^{2}+\left(\frac{\sigma_{g\times e}^{2}}{ny}\right)+\left(\frac{\sigma_{e}^{2}}{ny\times nr}\right)$$

Where *H*^2^ is the broad sense heritability, $\sigma_{g}^{2}$ is genotypic variances, $\sigma_{g\times e}^{2}$ is variance for genotype and environment interaction, *ny* number of years and *nr* number of replications”. Pearson’s correlation coefficients (r) noted to determine the association among studied traits through the SPSS ver.23 [34] under observed environments.

### Genotyping

Single accession was seeded in a polythene bag. Fresh 15-day-old wheat seedling leaf used for DNA isolation follow to the CIMMYT Manual of Molecular Genetics procedures [35]. DNA of respective accessions (70–100 ng/μl) stored in a 96-well plate and sent for genotyping to CapitalBio® in Beijing, China with a high-density Illumina 90,000 Infinium SNPs array (Wang et al. 2014). The genomes-wide positions of SNPs and genetic distance (cM) located on each chromosome were based on developed genetic map of bread wheat used in current experiment [36]. When analyzing data, monomorphic SNPs, missing values more than 20%, minor alleles and allelic frequency less than 5% were excluded.

The article "Genome-wide association mapping for high temperature tolerance in wheat through 90k SNP array using physiological and yield traits" was retracted in 2023. Reasons: a conflict of interest; concerns about the peer review; concerns about the authorship.

### Population structure

Bayesian grouping practice was used with SNP to rank cluster of genetically similar accessions using STRUCTURE v.2.3 [37]. Burn-in iterations of 10^4^ cycle and admixture modal selection have been used in this study. An ad-hoc web based method “Structure Harvester v0.6.93” was experienced obtaining high values or peak of ‘‘K” for the confirmation to identify the STRUCTURE results [38]. We select the K value ranged from 1 to 10 and 6 independent runs to accomplish the consistent effect.

### GWAS analysis

The GAPIT packages were applied to perform association mapping of studied attributed in RStudio [39]. This tool has been used with modal selection preferences to checked the dependability of the outcome [40]. Through this tool, the unconventional statistical methods implemented like compressed mixed linear modal (CMLM) and CMLM-base genome prediction selection and calculate the false discovery rates (FDR) [40, 41]. Threshold level for associated markers as significance (p-values) was restrained at 10^−3^ or more [7] after Bonferroni adjustment (P = 1/n, n = total numbers of SNPs) [42]. To determine the relevance of the applied model for GWAS, quantile-quantile (QQ) plot was derived among the observed and expected log10(*P*) value [19, 40]. Overall, 32,141 of the 81,000 functional iSelect beads chip analyses visually displayed polymorphic and noticed on the published genetic map [36].

## Results

### Phenotypic evaluation

In the current experiments, ANOVA of physiological and yield traits for 96 spring wheat genotypes exhibited significant effects on phenotype variability (P < 0.01). Studied attributes exhibited highly significant influence between examined genotypes as shown in S2 Table in S1 File. Broad-sense heritability of the considered traits was also measured (S2 Table in S1 File). The high heritability was detected for grain yield per plant (77.8%) and 1000-grain weight (76.4%) under heat stressed conditions. Canopy Temperature at vegetative stage and canopy temperature at grain filling stage displayed the heritability values 58.3% and 67.2% respectively under normal conditions while under heat stressed conditions the heritability was 61.3% and 64.4% respectively. The FLA showed the heritability as 71.9% and 68.5% in non-stressed and heat stressed condition respectively. The 72.2% and 59.6% heritability values were also noted for DH and DM respectively under non-stressed conditions, while 70.1% and H^2^ = 61.6% respectively under heat stressed conditions. Descriptive statistics data of studied characters in normal and heat stressed condition base on averaged data overs year have given in S3 Table in S1 File. Averaged value of FLA was 33 cm^2^ and 28 cm^2^ under normal and heat stressed conditions, respectively. The CMT had mean values 57% under normal conditions while in heat stress conditions as 48% in this study. The CTV and CTG exhibited mean performance as 35 and 28 under normal conditions, while, it was 27 and 30 under heat stressed condition, respectively. Day to headings and day to maturity was 90 days and 112 days under normal conditions while in heat stress conditions it changed as 81 days and 102 days respectively. Mean values of TGW was 73g and 31g in normal and heat stressed conditions, respectively. Mean values of GYP was 22g and 16g in normal and heat stressed conditions, respectively. Correlation coefficient of physiological and yield traits based on data average over year in normal and heat stressed conditions presented in Table 1. Highly significant correlations were recorded by canopy temperature at vegetative stage and grain filling stage with yield and yield related attributes. Significant positive association of FLA with grain yield per plant and thousand-grain weight was observed. Day to heading and thousand-grain weight exposed highly significant correlation with all other traits (Table 1). Under high temperature stress, correlation of CMT was positive and highly significant with yield related indices. Highly significant correlation of physiological and yield attributes was observed under both environments. The CTV was significantly associated with FLA, CMT, TGW and GYP in both environments.

The article "Genome-wide association mapping for high temperature tolerance in wheat through 90k SNP array using physiological and yield traits" was retracted in 2023. Reasons: a conflict of interest; concerns about the peer review; concerns about the authorship.

**Table 1:** Correlation coefficients of physiological and yield traits based on data average over year in normal and heat stress conditions.

Traits	Environment	FLA	CMT	CTV	CTG	DH	DM	TGW
**CMT**	N	0.58**						
	H	0.53**						
**CTV**	N	0.51**	0.47**					
	H	0.49**	0.59**					
**CTG**	N	0.48**	0.42**	0.48**				
	H	0.46**	0.46**	0.46**				
**DH**	N	0.49**	0.34*	0.54**	0.56**			
	H	0.47**	0.36*	0.51**	0.52**			
**DM**	N	0.55**	0.38*	0.59**	0.59**	0.77**		
	H	0.52**	0.33*	0.55**	0.48**	0.69**		
**TGW**	N	0.79**	0.52**	0.70**	0.61**	0.62**	-.43**	
	H	0.71**	0.51**	0.68**	0.54**	0.58**	-.47**	
**GYP**	N	0.84**	0.61**	0.71**	0.66**	0.68**	-.45**	0.81**
	H	0.79**	0.58**	0.66**	0.61	0.63**	-.44**	0.74**

### Population structure

Based on the STRUCTURE algorithm, the second order probability (*Δk*) was calculated from structure harvester, which exhibited maximum values when the given k (the numbers of sub-population base on the modal, K = 4) was four (S1 Fig in S1 File). Delta K showed only the highest clustering levels and numbers of subpopulation in main populations. In S2 Fig in S1 File the results obtained from STRUCTURE analyses and different colors showed the indication of different population. The similar results already published of genotypic data but associated with different traits. From these results, total 12 genotypes (G1-G10, G27- G28) fall in the same group and are considered as the first group. Only 14 accessions (G11-G22, G29-G30) were categorized in the second group. Overall 39 genotypes from G34 to G72 considered in third group. Genotypes G31, G32 and G33 contained mixed genetic material of the second and the third group. Seventeen accessions from G73 to G89 categorized in the fourth group. Genotypes G90, G91, G92, G93, G94, G95, and G96 also exhibited the collective genetic material of third and fourth groups.

The article "Genome-wide association mapping for high temperature tolerance in wheat through 90k SNP array using physiological and yield traits" was retracted in 2023. Reasons: a conflict of interest; concerns about the peer review; concerns about the authorship.

### Genome-wide MTAs for studied attributes

In the present experiment, 32,141 high density SNPs were assessed from the Illumina iSelect SNP 90K array to detect SNP linked with physiological and yield attributes. The markers traits association for these traits were observed and 320 SNPs were significant linked to the traits, out of them 169 and 151 MTAs found in normal and heat stressed environments, respectively, at *P ≤* 0.0001 threshold level (S4 and S5 Tables in S1 File). Manhattan plots (Figs 1–4) presenting the sites of significant SNPs at -log10(p) ≤ 3 which associated with the specific characters and examined environments. The quantile-quantile (QQ) plots of p-values were created (S3–S18 Figs in S1 File) to confirm the results of Manhattan plots as mentioned in these figures. The Y-axis was the observed negative base 10 logarithm of the p-values, and the X-axis showed the expected observed negative base 10 logarithm of the p-values under the assumption that the p-values follow a uniform (0, 1) distribution. The dotted lines show the 95% confidence interval for the QQ plot under the null hypothesis of no association between the SNP and the trait.

**Fig 1:** Manhattan plot of Flag leaf area (FLA) in normal (**A**), heat stressed (**B**) conditions and Cell membrane thermostability (CMT) in normal (**C**) heat stressed (**D**) conditions. These figures exhibiting the position of significant SNPs and -log10(p) linked with specific traits in normal and heat stressed conditions.

**Fig 2:** Manhattan plot of Canopy Temperature at vegetative stage (CTV) in normal (**A**), heat stressed (**B**) conditions and Canopy Temperature at grain filling stage (CTG) in normal (**C**) heat stressed (**D**) conditions. These figures exhibiting the position of significant SNPs and -log10(p) linked with specific traits in normal and heat stressed conditions.

The article "Genome-wide association mapping for high temperature tolerance in wheat through 90k SNP array using physiological and yield traits" was retracted in 2023. Reasons: a conflict of interest; concerns about the peer review; concerns about the authorship.

**Fig 3:** Manhattan plot of Days to heading (DH) in normal (**A**), heat stressed (**B**) conditions and Days to maturity (DM) under normal (**C**), heat stressed (**D**) conditions. These figures exhibiting the position of significant SNPs and -log10(p) linked with specific traits in normal and heat stressed conditions.

**Fig 4:** Manhattan plot of thousand grain weight (TGW) in normal (**A**), heat stressed (**B**) conditions and Gain yield per plant (GYP) in normal (**C**), heat stressed (**D**) conditions. These figures exhibiting the position of significant SNPs and -log10(p) linked with specific traits in normal and heat stressed conditions.

### Morphological and physiological traits

#### Flag leaf area (FLA)

Twenty-two markers exhibited high significant associations with flag leaf area which situated at chromosome, 2A, 3A, 5A 3B, 4B, 7B, 1D, 3D and 5D (Fig 1A) in normal condition. The loci associated with this attribute exhibited an explained phenotypic variation from 12.68% to 19.83% of the total phenotypic variation. Significant MTAs for this trait were dispersed overall three genomes, as well as 3 SNPs from A-genomes, seven from B-genomes and twelve from D-genomes. The marker (*BS00045521_51*) explain the high values of trait variation (19.83%) on chromosome 1A at 341.14cM while the marker (*Ra_c11906_1618*) from chromosome 1D at 172.13cM explain the low value (12.68%) of trait variation of flag leaf area under normal conditions (S4 Table in S1 File). Under heat stress conditions, nineteen SNPs were strongly linked with flag leaf area on chromosome 3A, 5A, 7A 1B, 2B, 3B and 6B (Fig 1B). Total phenotypic variation revealed by associated linked SNPs ranged from 17.10% to 37.15%. Significant MTAs for this trait were located on two wheat genomes, counting 7 SNP from A-genome, 12 from B-genome and none of the significant MTAs from D genome. The marker (*Kukri_c55051_414*) had maximum PVE (37.15%) on chromosome 5A at 68.2cM whereas the marker (*RAC875_c1036_897)* on the 6B chromosome (S5 Table in S1 File) explained the least proportion 17.10% of the trait phenotypic variability at 386.86cM position.

#### Cell membrane thermo-stability

In normal experimental conditions, nine SNPs are linked with cell membrane thermostability out of these, four are situated at chromosome 3D and the remaining were at chromosome 1B, 2B, 3A, 4A and 7B (S4 Table in S1 File). These 9 MTAs explain 24.13% to 32.35% of the variation in this trait. Significantly MTAs for this trait were distributed on all wheat genomes, including 2 SNPs from the A-genome, three from the B-genome and four from the D-genome (Fig 1C). The marker (*Tdurum_contig100702_265*) explain maximum phenotypic trait variation (32.35%) on chromosome 4A at 542.67cM while the marker (*tplb0028p08_626*) on chromosome 3D at 13.29cM explain a low value (24.13%). Under heat stress conditions, 27 MTAs explain phenotypic variation ranged from 19.21% to 41.09% in this attribute. These significantly associated SNPs were perceived at chromosomes 1A, 3A, 4A, 5A, 7A, 1B, 2B, 3B, 4B, 5B, 7B, 2D, 3D, 5D and 7D (Fig 1D). The marker (*Excalibur_c53131_187*) explained highest phenotypic trait variation on chromosome 3A at 276.05cM while the marker (*RFL_Contig1319_507*) on chromosome 3B at 268.75cM explained low value (S5 Table in S1 File). Associated MTAs for this trait were dispersed on the overall genome, including ten SNPs from A-genome, nine from B-genome and eight from D-genome under heat stressed conditions.

The article "Genome-wide association mapping for high temperature tolerance in wheat through 90k SNP array using physiological and yield traits" was retracted in 2023. Reasons: a conflict of interest; concerns about the peer review; concerns about the authorship.

#### Canopy temperature at vegetative stage (CTV)

In the non-stressed environments, canopy temperature at vegetative stage (CTV) was highly correlated with 30 MTAs, out of them, seven MTAs were situated at each chromosomes 2D and 7B, three MTAs on each chromosome 4B and 5A, two MTAs on each chromosomes 3B and 7A while one MTA associated on each of chromosome 1A, 1B, 2B, 6B, 5D and 7D (Fig 2A). They explain the phenotypic variation from 18.12% to 34.98%. Significantly MTAs for CTV were dispersed on all wheat genomes, including 7 SNPs from the A-genome, fourteen from the B-genome and nine from the D-genome (S4 Table in S1 File). The marker (*Tdurum_contig79608_369*) exhibited more phenotypic variation (34.98%) on chromosome 1A at the position of 312.46cM, while the marker (*BS00079076_51*) showed least phenotypic variation (18.12%) at chromosome 7B at the positions of 296.21cM in normal conditions. In heat stressed conditions, fourteen MTAs explained phenotypic variation ranged from 24.94% to 37.40% in this attribute. Three SNPs were detected at chromosome 6D, two at each of 1B, 3D, 4A, 5A, while on at 7B (Fig 2B). The marker (*BS00010616_51*) explained more phenotypic trait variation (37.40%) on chromosome 7B at 186.24cM, while the marker (*GENE-4153_101*) on chromosome 6D at 180.23cM explain minimum value (24.94%) under heat stress conditions (S5 Table in S1 File). Significantly MTA for this trait was dispersed on the whole genome, counting 4 SNP from the A-genome, three from the B-genome and seven from the D-genome.

#### Canopy temperature at grain filling stage (CTG)

Under non-stresses conditions, twenty-three markers exhibited highly significant associations with this attribute which were found on chromosomes 1A, 4A, 5A, 7A, 1B, 2B, 3B, 7B, 1D, 2D, 3D, 5D, 6D and 7D in this study (Fig 2C). Associated loci of canopy Temperature at grain filling stage presented phenotypic variability explain (PVE) from 20.58% to 37.86% of the total phenotypic variability. These loci were dispersed among the whole wheat genome, including 8 SNPs from the A-genome, also 8 from the B-genome and seven from the D-genome. The marker (*Tdurum_contig48049_705*) explain the highest value of trait variation (37.86%) on chromosome 4A at 160.42cM while the marker (*Kukri_c78263_296*) from chromosome 6D at 118.9cM explain the least value (20.58%) of trait variation of this character under normal conditions (S4 Table in S1 File). Under heat stress conditions, nineteen SNP were linked with CTG on chromosome 2A, 2D, 4B, 5B, 6B and 7A (Fig 2D). Total phenotypic variation by linked marker ranged from 22.32% to 28.92% and also dispersed in three wheat genomes, including 8 SNPs from the A-genome, nine from the B-genome and two from the D-genome. The marker (*BobWhite_c25703_160*) on chromosome 7A at 687.47cM had more PVE (28.92%), while the marker (*Kukri_rep_c69515_183*) on the 5B chromosome explained the minimum proportion (22.32%) of the trait PVE at 199.86cM position (S5 Table in S1 File).

The article "Genome-wide association mapping for high temperature tolerance in wheat through 90k SNP array using physiological and yield traits" was retracted in 2023. Reasons: a conflict of interest; concerns about the peer review; concerns about the authorship.

#### Days to heading (DH)

In non-stressed conditions, this trait was highly associated with nineteen markers. Four significantly MTAs linked with DH were perceived on chromosome 7B, 2 MTA on each 1B, 3D, 5A and 1 on each 1A, 4A, 7A, 2B, 3B, 1D, 2D, 5D and 7D as mentioned in Fig 3A. These 19 DH related markers explained 21.14% to 37.86% of the variability in this attributes (S4 Table in S1 File). The marker *Tdurum_contig48049_705* explained the maximum phenotypic variability (73.86%) on chromosome 4A at position 160.42cM for this trait. The marker namely *TA001877-0445* exhibited the minimum phenotypic variation which located at chromosome 3D with position 263.93cM in this studied trait. Associated MTAs dispersed on A, B and D genome, including five SNPs from the A-genome, eight from the B-genome and six from the D-genome. In heat stressed conditions, 24 significant SNPs were positively associated with DH counting 7 markers situated on chromosome 4B, 5 markers situated on chromosome 3B, 4 markers situated on chromosome 3D, 3 markers situated on chromosome 6A and 2 markers situated on chromosome 2B, while 1 SNPs on each chromosomes 1B, 5A and 6B (Fig 3B). These markers explained 19.02% to 39.13% of the phenotypic variation for DH in heat stress conditions. The SNP *Excalibur_rep_c111191_119* on chromosome 3D at 379.04cM distance revealed a highest phenotypic variation 39.13%, while the marker *IAAV1653* on chromosome 3B at 269.78cM distance indicated minimum phenotypic trait variation (S5 Table in S1 File). Four SNPs observed on A-genome, sixteen from the B-genome and seven from D-genome in heat stressed conditions.

The article "Genome-wide association mapping for high temperature tolerance in wheat through 90k SNP array using physiological and yield traits" was retracted in 2023. Reasons: a conflict of interest; concerns about the peer review; concerns about the authorship.

#### Days to maturity (DM)

Days to maturity (DM) was highly linked with twenty-seven markers in non-stressed environments. Significantly associated MTAs were perceived on chromosome 1A, 3A, 4A, 5A, 7A,1B, 2B, 3B, 4B, 7B, 1D, 2D, 3D, 5D, 6D and 7D (Fig 3C) for this attribute. These sixteen DM related markers explain the total phenotypic variation 18.35% to 36.38% (S4 Table in S1 File). The marker *Tdurum_contig48049_705* on chromosome 4A at 160.42cM explained more phenotypic variation (36.38%), while the marker *Kukri_rep_c105589_73* on chromosome 1A at 261.32cM explain the least values (18.35%) under normal conditions. Significant MTAs for this trait were dispersed on A, B and D genomes, including 10 SNPs from each A and B-genomes while seven from the D-genome under normal conditions. Under heat stressed conditions, twenty significant SNPs were strongly linked with DM as well as four markers detected on chromosome 7B, 2 SNPs on each chromosomes 1A, 1B, 3D, 5A, and one on each 4A, 7A, 2B, 3B, 1D, 2D, 5D and 7D as mentioned in Fig 3D. The marker *Tdurum_contig48049_705* explain the maximum trait variation (35.71%) on chromosome 4A at 160.42cM, while the marker *Tdurum_contig42214_2997* on chromosome 2B at 285.18cM explained the least values (20.00%) under heat stress conditions. Six associated markers were observed from the A genome, 8 SNPs from B-genome and 6 from the D-genome under heat stress conditions. These markers explained 20.00% to 35.71% of the phenotypic variation in days to maturity under heat stress conditions (S5 Table in S1 File).

#### 1000-grain weight (TGW)

Total twenty-two significant MTAs were observed for the TGW in normal conditions. Out of them, four MTAs were recorded at chromosomes 4B, 3 MTAs on chromosome 3D, 2 MTAs on each of chromosome 4A, 5A, 6B, 7D while one at each of 3A, 7A, 1B, 2B, 5B, 7B and 3D (Fig 4A). Phenotypic variability designated by these MTAs varied from 17.47% to 31.26% for this attribute. The marker *Excalibur_c53131_187* explain the maximum phenotypic variation (31.26%) on chromosome 3A at 276.05cM, while the marker *Kukri_c56014_275* on chromosome 4A at 425.2cM explain least values (17.47%) under normal conditions (S4 Table in S1 File). Under heat stress condition, sixteen significantly associated SNPs were positively linked with TGW. These significantly associated SNPs were situated at different chromosomes. Out of them, 11 were situated at chromosomes 2D, 3 were observed at 4D while the one on each 4A and 6D (Fig 4B). The marker *RAC875_c6138_1112* explained more phenotypic trait variation on chromosome 6D at 63.55cM, while the marker (*Kukri_c63505_174*) on chromosome 2D at 110.64cM explained less phenotypic variation under heat stress conditions (S5 Table in S1 File). These SNPs had 16.37% to 24.23% variation in TGW under heat stressed conditions.

The article "Genome-wide association mapping for high temperature tolerance in wheat through 90k SNP array using physiological and yield traits" was retracted in 2023. Reasons: a conflict of interest; concerns about the peer review; concerns about the authorship.

#### Grain yield per plant (GYP)

Seventeen MTAs were observed for GYP in normal conditions, located at chromosome 2A, 4A, 5A, 1B, 2B, 4B, 5B, 6B, 7B and 7D (Fig 4C). These MTAs explained 20.57% to 33.64% of the variation and dispersed on A, B and D genomes, including, six MTAs at A-genome, ten at B-genome and one at D-genome. The marker *RAC875_c3397_1492* presented highest phenotypic variation on chromosome 2A at the position of 402.04cM, while the marker (*Kukri_c18857_260*) showed the least phenotypic variation on chromosome 2B at the position of 351.23cM in non-stressed conditions (S4 Table in S1 File). Twelve significant loci were seeming for this character in heat stressed conditions (Fig 4D). Out of them, two associated SNPs located on chromosome 5A, while one on each chromosomes 2A, 3A, 7A, 2B, 3B, 7B, 4B, 3D, 5D and 7D explaining 22.47% to 33.92% variation for GYP under heat stress conditions. The marker *BS00072620_51* explain high trait variation on chromosome 2B at 124cM, while the marker *Kukri_rep_c101206_312* at chromosome 5A at 78.63cM explained less variation in heat stressed conditions. These MTAs were dispersed on A, B and D genomes, including, five MTAs at A-genome, four at B-genome and three at D-genome in heat stressed conditions (S5 Table in S1 File).

### Genome-wide multiple traits loci associations

Trait-wise maximum number of MTAs were recognized for CTV (30) followed by DM (27), CTG (23), FLA (22), TGW (22), DH (19) GYP (17) and CMT (9) under normal conditions. Under heat stressed conditions, high number of MTAs was perceived for CMT (27) followed by DM (20), FLA (19), CTG (19), CTV (14), TGW (16) and GYP (12) in the present study (Table 3). Chromosome-wise, maximum MTAs were observed on chromosomes 7B (22), 4B (15), 5A (13), 2D (13) followed by 1D (11), 1B (10), 2B (9) and 7A (9) in non-stress conditions. The A genome relatively exhibited a low number of MTAs (47), but the B genome contained more MTAs (70), and the D genome have (52) MTAs in non-stressed conditions in the present study. The chromosome-wise observing, MTAs recorded on chromosomes more 2D (16), than 5A (13), 7A (13), 3B (11), 4B (11) and 3D (10) followed by 2B (10), 7B (8) and 7D (7) under heat stressed conditions. The B genome contained lowest MTAs (61), while the A and D genomes had same number (45) of MTAs under heat stressed conditions in the current experiment (Table 3).

Observing the A genome, associated markers (*BS00065292_51* and *Excalibur_c13242_1178*) showed the least phenotypic variability 13.99% and 17.27% on chromosomes 5A and 3A having the position of 400.13cM and 279.61cM were considerably linked with flag leaf area under non-stressed and heat stressed condition, respectively (S4 and S5 Tables in S1 File). Highest phenotypic variation 37.86% and 41.09% happened in A genome characterized by the significantly associated markers *Tdurum_contig48049_705* and *Excalibur_c53131_187* from chromosomes 4A and 3A with the position of 160.42cM and 276.05cM were associated with DH and CMT in normal and heat stressed environments, respectively. The significantly associated markers, namely *RFL_Contig3563_1130* and *RAC875_c1036_897* were correlated with flag leaf area in the B genome from chromosome 4B (199.73cM) and 6B (386.86cM) explain the minimum phenotypic traits (13.08% and 17.10%) variation in normal and heat stressed conditions, respectively. In genome B the significant SNPs (*BS00013824_51* and *BS00010616_51*) observed the maximum trait variation 32.73% and 37.40% from chromosomes 1B and 7B with the position of 208.49cM and 186.24cM for CTV under both examined conditions (S4 and S5 Tables in S1 File). The significant SNPs namely, *Tdurum_contig1015_131* and *Excalibur_rep_c111191_119* located on chromosomes 3D (292.51cM) and 3D (379.04cM) were linked with DH in D genome exhibiting maximum phenotypic variation 36.51% and 39.13% in non-stressed and heat stressed conditions, respectively (S4 and S5 Tables in S1 File). The minimum phenotypic trait variability12.68% and 16.37% occurred in the D genome described by the markers *Ra_c11906_1618* and *Kukri_c63505_174* on chromosomes 1D and 2D with the position of 172.13cM and 110.64cM were linked with FLA and TGW in normal and heat stressed environments, respectively.

The article "Genome-wide association mapping for high temperature tolerance in wheat through 90k SNP array using physiological and yield traits" was retracted in 2023. Reasons: a conflict of interest; concerns about the peer review; concerns about the authorship.

Pleiotropic locus *BobWhite_rep_c61300_88* on chromosome 7B at 206.22cM was significantly linked with yield and heat stress-related attribute like DH, CTG and DM (S4 Table in S1 File). The examined characters like DH, CTG, DM and GYP was influenced by a pleiotropic locus *Excalibur_c27873_266* on chromosome 1D at 268.67cM under normal conditions as shown in S4 Table in S1 File. Under heat stress conditions, pleiotropic loci namely *wsnp_Ex_rep_c66522_64795143* correlated with CTV and DM was identified on chromosome 2D. Pleiotropic loci *BobWhite_c836_422 and BS00010616_51* were associated with CTV and DM, situated at chromosomes 5D and 7B having the position of 162.12cM and 186.24cM, respectively, in heat stressed environments (S5 Table in S1 File). Another pleiotropic locus reported in this study, *D_GA8KES401BNLTU_253*, *Kukri_rep_c87210_361* and *Tdurum_contig1015_131* on chromosomes 1B, 5A and 3D at the positions 243.59cM, 77.82cM and 292.51cM, respectively, were associated with examined attributes in both environments (S2 and S5 Tables in S1 File). Multi-trait loci for physiological and yield characters were predicted on chromosomes 4A, 5A, 1B, 7B, 2D and 3D in studied environments.

## Discussions

### Phenotypic evaluation

Enhancing of wheat grain yield is an excessive precedence of wheat researchers with a purpose to meet growing needs worldwide. Results of the present experiment showed that highly significant differences occurred between genotypes and environmental conditions, indicating the presence of variations and environmental effects on the behavior of genotypes for the examined traits (S2 Table in S1 File). The similar information have been reported previously [14, 33, 43]. Heritability estimations provide the evidence about the amount of which a genetic trait is to be transferred to succeeding generation. High heritability was stated in the examined attributes, like TGW (77.8%), followed by DH (72%), FLA (71.9%), CTG (67.2%) and DM (59.6%) which indicated (S2 Table in S1 File) the additive genetic effect on inheritance, and the selections may be effective in early generation for these attributes. Mean values of grain yield/plant was 22g and 16.g in non-stress and heat stress conditions, respectively. Various genotypic variability in response to heat stress and adversative impact on the performance of genotypes earlier observed by wheat researchers [44]. It has also been found that in wheat cultivation, the highly reduction in grain developments due to heat stress conditions during anthesis and post-anthesis phases [5, 10] which in due course lessen the total grain yield. Correlation coefficient based on average data over year in non-stressed and heat stressed conditions also analyzed in studied attributes (Table 1). The CTV and CTG showed highly significant correlation. Previously wheat scientists [45] found significant results and showed accordance with our results that. Some researchers [6] observed positively and non-significant associations of CTV and CTG with GYP that show contradiction with current findings due to having different germplasm and different environmental conditions. Wheat breeders [46] also reported similar positive significant association of thousand grain weight with grain yield per plant in wheat. Under high temperature stress, correlation of CMT was positive and highly significant with yield and related traits. Significant negative correlation of DM with yield traits was observed in this study. Under heat stress, Flag leaf area showed positive significant correlations with yield traits. The CTV showed positive correlation with FLA, CMT, TGW and GYP in both environments (Table 1). Previously reported results [47] also show positive significant correlation of TGW with GYP in heat stress that show accordance with our results. Few motives are correlated with the various pathways because high temperature stress alter the pathways, which caused yield losses in wheat [48]. Grain yield exhibited negatively association with days to maturity in the current study, signifying that early maturing plant had maximum production than the late maturing plant in heat stress environments [5]. The yield related traits and physiological traits like FLA, CMT, CTV, CTG, DH, TGW and GYP exhibited positively correlation in normal and heat stress conditions. The selections of these attributes will be beneficial [27] for further breeding programs. CMT and other physiological attributes already used to select heat tolerant varieties [13]. Among the genotypes with different behavior in normal and heat stress condition, the best performing genotypes were considered as heat stress tolerant. By using observation, the six heat-tolerant wheat genotypes (G1, G6, G11, G16, G21, and G39) were classified from the studied germplasm as shown in Table 2.

The article "Genome-wide association mapping for high temperature tolerance in wheat through 90k SNP array using physiological and yield traits" was retracted in 2023. Reasons: a conflict of interest; concerns about the peer review; concerns about the authorship.

**Table 2:** Best performance wheat genotypes in normal and heat stress condition based on averaged data over year.

Trait	Normal	Heat stress
FLA	G16 followed by G11, G21, G6, G1 and G39	G1 followed by G6, G21, G11, G39 and G16
CMT	G6 followed by G39, G11, G16, G21 and G1	G11 followed by G6, G39, G6, G21 and G1
CTV	G11 followed by G16, G21, G1, G6 and G39	G1 followed by G16, G21, G11, G39 and G6
CTG	G16 followed by G1, G6, G11, G39 and G21	G16 followed by G11, G21, G6, G39 and G1
DH	G1 followed by G11, G16, G21, G6 and G39	G16 followed by G21, G6, G39, G11 and G1
DM	G39 followed by G16, G1, G6, G21 and G11	G6 followed by G11, G21, G39, G16 and G1
TGW	G21 followed by G16, G1, G39, G6 and G11	G16 followed by G11, G21, G39, G6 and G1
GYP	G11 followed by G1, G6, G16, G39 and G21	G21 followed by G11, G6, G39, G6 and G16

### Population structure

The Bayesian approach implemented in the STRUCTURE version 2.3 statistical software package was applied to evaluate the genetic structures of 96 accessions. This methodology was also used earlier in the wheat breeding program by numerous researchers and the descriptive results were obtained.

In wheat breeding program, these methods have also been applied by numerous wheat scientists [5, 7]. The STRUCTURE analysis recommended discrepancies between 96 genotypes representing genetic similarity within groups and genetic dissimilarities among the groups. Mainly, the results practically deliberated on the origin and pedigree record already identified for the wheat genotypes. [10, 15]. Genotypes contained varied genetic makeup would be nominated for desired combination to develop multiple and significance indices to obtained maximum yield.

The article "Genome-wide association mapping for high temperature tolerance in wheat through 90k SNP array using physiological and yield traits" was retracted in 2023. Reasons: a conflict of interest; concerns about the peer review; concerns about the authorship.

### Genome-wide marker traits associations

The effect of heat stress is usually described in many parts of the world due to climate change. In the present experiment, our objective was to determine genomic parts for different physiological and yield related attributes in heat stress conditions using a genome-wide associations approach. Genes and QTLs linked to examined attributes, were dispersed across twenty-one chromosomes designated by many scientists [7, 14]. Marker-trait association (MTA) examine diagnosed the relationship among a selected morphology and genetics variant inside a genome, which in the end apparent locus underpinning associated traits [49]. In the present experiment, 32,141 polymorphic SNPs from a high density 90,000 Illumina iSelect array [36] were observed to detect linked SNPs with physiological and yield characters [33]. Marker-trait associations (MTA) for these characters in non-stressed and heat stressed environments were detected. The quantile-quantile (QQ) plot between the detected negative base 10 log of the *P*-value and expected negative base 10 log of the *P-*value with the assumptions that the *P*-value monitor a constant [0,1] scattering was observed as well. The dotted line showed the 95% confidence intervals for the QQ-plots in the null hypothesis of zero (0) correlation among SNPs and the studied traits (S3-S18 Figs in S1 File). This study allowed us to identify important genomic regions carrying some important genes associated with studied traits. The flag leaf area of the wheat plant is an important character and directly influences on yield because a greater area enables us to produce photosynthates in higher amounts, which are translocated in seed to increase their yield. Earlier research was in line with current results they reported MTAs for FLA on chromosome 1B, 4D, 5A, 6B, 7D using a wheat recombinant inbred line (RIL) population under normal and different water stressed conditions [19]. MTAs for FLA were distributed on overall 3 genomes, three MTA at A-genome, seven at B-genome and twelve at D-genome in normal conditions in this study. Previously researchers found the MTAs for FLA on chromosomes, 5A, 1B, 6B, 4D and 7D which were similar to our studied results in wheat crop [50]. Wheat researchers used the high-density SNP genetic linkage maps in wheat genotypes and identify the 13 chromosomes region to be linked with flag leaf area having 3.33–26.13% of trait variability [51]. MTAs were situated on chromosomes 4A, 4B and 5B, with QTLs for canopy temperature (4A and 4B) for day to headings and day to maturity (5B) also observed by wheat scientists [14]. The significantly MTAs for CMT were dispersed across A, B and D genome, including 10 SNP at A-genome and 9 SNP at B-genome and eight at D genome in heat stressed condition in this study. Earlier scientists evaluated a heat stressed condition in wheat and reported the high temperature tolerance QTL qDHY.3BL in ~1Mbp on chromosomes 3B, containing 22 accountable genes for CMT trait [18].

The article "Genome-wide association mapping for high temperature tolerance in wheat through 90k SNP array using physiological and yield traits" was retracted in 2023. Reasons: a conflict of interest; concerns about the peer review; concerns about the authorship.

Previously scientists [52] recognized eight QTLs cluster linked with heat stress tolerance on chromosomes 1B, 2B, 2D, 4A, 4B, 4D, 5A, and 7A, which suggesting that the fine mapping techniques may be useful to recognize the gene in these genomic parts (S5 Table in S1 File). Significant MTA for DH were dispersed across all genomes including five SNP in A-genome and eight in B-genome and six in D genome in this study. Up to the present time, determination of QTLs/genes in wheat for heat tolerant has been is mostly directed at the time of grain filling stage [44]. This research diagnosed numerous predominant and minor QTLs for vegetative and reproductive level developments on various wheat chromosomes. For example, 5 QTLs for heat tolerance in wheat have been detected on chromosomes 1B, 1D, 2B, 6A and 7A [15]. Likewise, two QTLs for heat tolerance were observed on chromosomes 2B and 5B in a map population of spring wheat [7]. Yet in other studies, QTLs have been found for heat tolerance during the grain filling phase on different chromosomal regions, like 1A, 1B, 2B, 3B, 5A and 6D [44]. Additionally, QTLs were linked with physiology and yield traits have been found on chromosomes 2A, 3A, 4A, 6A, 6B and 7A [12].

Consistent with the previous findings using chromosome replacement lines, numerous QTLs controlling heat stressed tolerance were situated on chromosomes 3B. A previous report [44] recognized an important QTL regions on the 3B chromosome in wheat linked with the heat sensitivity index of the yield indices. Two key QTLs on chromosome 3B for canopy temperature and yield per plant have been observed [53] by studying a set of 255 wheat advanced lines. Earlier studies [54] also recorded QTLs controlling canopy temperature which located on chromosomes 3B. Additionally, [18] recorded heat tolerant linked QTLs, *qDHY*.*3BL*, in an ~1 Mbp interval on chromosomes 3B, which confined twenty-two genes in wheat.

Highly phenotypic traits relation could be defined in relative to the direct or indirect effect of a trait on another trait. Within the genomes, those traits can be managed via way of means of pleiotropic loci. It is demonstrated by the occurrence of several MTAs in which a gene will display a pleiotropic influence on multiple related traits [27]. MTA for TGW sixteen significantly associated SNPs were positively linked with 1000-grain weight. These significantly associated SNPs were situated at various chromosomes. Out of them, 11 were situated at chromosomes 2D, 3 were observed at 4D while the one on each 4A and 6D in this study (S18 Fig in S1 File). Stable genomic parts for TGW have commonly been recognized on chromosomes 5A, 3B and 5B that impact TGW in several population of wheat with association mapping study described by wheat researchers [55]. Remarkably, chromosome 5B stated by wheat scientists [56] that harbor a region regulating several yield-associated traits was identified which have genomic regions associated with studied traits in current experiment. MTA controlling GYP found on chromosomes 1A, 4B, 6B, and 7D [56]. The MTA on 5A was associated with GYP in non-stressed conditions defined by earlier researchers [5]. Similarly, Edae et al. [57] designated significantly associated MTAs for grain yield per plant at chromosomes 4A, 1B, 5B and 2B. Furthermore, Lozada et al. [58] also stated MTAs for this characters on chromosomes 5A, 1B, 2B and 4B. These associated MTAs were particular to various environmental conditions signifying dynamic nature of genetics consistent to wheat yield [58]. The maximum numbers of MTAs genome-wise and chromosome-wise are given in Table 3.

The article "Genome-wide association mapping for high temperature tolerance in wheat through 90k SNP array using physiological and yield traits" was retracted in 2023. Reasons: a conflict of interest; concerns about the peer review; concerns about the authorship.

**Table 3:** Significant MTAs under normal and heat stressed conditions.

Significant MTAs					
Genome-wise and Chromosome-wise			Traits-wise		
Genome	Normal	Heat stress	Traits	Normal	Heat stress
A Genome	Total 47 MTAs (1A = 8, 2A = 5, 3A = 5, 4A = 7, 5A = 13, 7A = 9)	Total 45 MTAs (1A = 3, 2A = 3, 3A = 5, 4A = 5, 5A = 13, 6A = 3, 7A = 13)	FLA	22	19
			CMT	9	27
			DH	19	24
B Genome	Total 70 MTAs (1B = 10, 2B = 9, 3B = 6, 4B = 15, 5B = 3, 6B = 5, 7B = 22)	Total 61 MTAs (1B = 7, 2B = 10, 3B = 11, 4B = 11, 5B = 4, 6B = 10, 7B = 8)	CTV	30	14
			CTG	23	19
D genome	Total 52 MTAs (1D = 11, 2D = 13, 3D = 12, 5D = 7, 6D = 2, 7D = 7)	Total 45 MTAs (1D = 1, 2D = 16, 3D = 10, 4D = 3, 5D = 4, 6D = 4, 7D = 7)	DM	27	20
			TGW	22	16
			GYP	17	12

### Genome-wide multiple traits loci associations

*Pleiotropic loci have seemed on chromosomes 4A, 5A, 7A, 1B, 2B, 3B, 4B, 6B, 7B, 1D, 2D, 3D, 7D which were associated with most of the studied attributes under normal conditions in the present study. Multi-trait-loci were seemed on chromosomes1A (DH, CTG, DM and CTV), 3A (FLA, CMT, TGW, DM and CTV), 4A (TGW, GYP, CMT, DH, CTG and DM), 5A (FLA, GYP, CTV, DH, CTG, DM, TGW), 7A (CTV, DH, CTG, DM and TGW), 1B (CTV, CMT, GYP, DH, CTG, DM and TGW), 2B (TGW, GYP, CTV, CMT, DH, CTG and DM), 3B (CTV, FLA, DH, CTG and DM), 4B (FLA, CTV, DM, GYP and TGW), 6B (GYP, TGW and CTV), 7B (CMT, DH, CTG, DM, CTV, TGW, GYP and FLA), 1D (DH, CTG, DM and FLA), 2D (CTV, TGW, DH, CTG and DM), 3D (TGW, CMT, FLA, DH, CTG and DM), 5D (DH, CTG, DM, FLA and CTV), 7D (CTV, TGW, GYP, DH, CTG and DM) in non-stressed condition. The Q gene located on chromosome 5A established the easy threshing of spike, plant height, spike length and emergence time of spike, and the pleiotropic effects of several yield related attributes like [59] Pleiotropic loci appeared on chromosomes 4A, 5A, 1B, 7B, 2D, 3D, 5D under heat stress conditions. Multi-trait loci have been identified on chromosomes 3A (GYP, FLA and CMT), 4A (CMT, CTV and DM), 5A (TGW, CTV, DM, FLA, GYP and DH), 7A (CTG, FLA, DM, CMT and GYP),1B (CTV, DM, FLA, CMT and DH), 2B (FLA, CMT, GYP, DH and DM), 3B (FLA, GYP, CMT, DM and DH), 4B (GYP, CTG, CMT and DH), 6B (CTG, DH and FLA), 7B (DM, CTV, GYP and CMT), 2D (CTG, CMT, TGW, CTV and DM), 3D (DH, CMT, GYP, CTV and DM), 5D (CTV, DM, CMT and GYP), 7D (CMT, GYP and DM) under heat stressed conditions (Table 3). Mainly QTL related with heat-stressed tolerance have been identified at chromosomes 1B, 2B, 2D, 4A, 4D, 5A, and 7A previously described by numerous researchers [7, 44, 52]. The distal regions of chromosome 7A and 7B are designated to contain QTLs for yellow pigmentation for grain, which are focused by Phytoene synthase1 (*PSY-1*) gene, the existence of this gene show the pleiotropic effect at 7B [60]. The* TaSnRK2 *gene resolute sucrose non-fermenting 1-related protein kinase located at chromosomes 4A and 4B. It has played an important role in responding against numerous environmental conditions and depict significance correlation with grain yield [61]. Wheat yield associated genes, such as* TaGW2-A1 *at 6A* TaTGW6-A1 *at 3A*, TaCwi *at 2A*, TaGS5-A1/TaGS-D1 *at 4A*, TaSus1 *at 7A and* TaSus2 *at 7B described by many scientists [62, 63].*A pleiotropic locus modified the appearance of numerous phenotypic traits, in this study, several pleiotropic loci have been documented. In normal conditions, pleiotropic locus *BobWhite_rep_c61300_88* on chromosome 7B at 206.22cM were significantly linked with yield and heat stress related attributes such as DH, CTG and DM. Another pleiotropic locus *Excalibur_c20796_395* at chromosome 7A on the positions 372.34cM was also associated with physiological and yield related traits in this study. The examined characters like DH, CTG, DM and GYP was influenced by a pleiotropic locus *Excalibur_c27873_266* on chromosome 1D at 268.67cM under normal conditions. The markers *Tdurum_contig42087_1199*, *Tdurum_contig46877_488* and *RAC875_c103017_302* on chromosomes 6B, 7B and 4B at 229.64cM, 178.15cM and 263.93cM respectively, showed pleiotropic effects for DH, CTG, DM and GYP under normal conditions as shown in S4 Table in S1 File. Pleiotropic loci *BobWhite_c836_422* and *BS00010616_51* were associated with CTV and DM, situated at chromosomes 5D and 7B with the position of 162.12cM and 186.24cM, respectively, in heat stress condition. Other pleiotropic loci *D_GA8KES401BNLTU_253*, *Kukri_rep_c87210_361* and *Tdurum_contig1015_131* on chromosomes 1B, 5A and 3D at the position of 243.59cM, 77.82cM and 292.51cM, respectively, showing the significance behavior with examined attributes in non-stressed and heat stressed environments. Herein, MTAs for physiological and yield related characters identified on chromosome 4A, 5A, 1B, 7B, 2D and 3D in both environments as given in Table 3. These MTAs would constitute a useful selection objective in wheat breeding scheme. As the intervals are still wide, fine genetic mapping will be essential to establish MTAs are a single locus with pleiotropic effects.

The article "Genome-wide association mapping for high temperature tolerance in wheat through 90k SNP array using physiological and yield traits" was retracted in 2023. Reasons: a conflict of interest; concerns about the peer review; concerns about the authorship.

## Conclusion

Heat stress showed adverse effects and declined grain yield in wheat. Positive association exists among physiological and yield attributes like FLA, CMT, CTV, CTG, DH, DM, TGW, and GYP in heat stressed environments. Therefore, the germplasm selection based on these traits would be fruitful in breeding for high temperature tolerant wheat genotypes. Under normal conditions, the markers *RAC875_c103017_302*, *Tdurum_contig42087_1199*, and *Tdurum_contig46877_488* and on chromosomes 4B, 6B and 7B at 263.93cM, 229.64cM, and 178.15cM respectively, were not only significantly associated with physiological and yield traits but also showed pleiotropic effects for DH, CTG, DM and GYP. The Markers *BobWhite_c836_422* and *BS00010616_51* on chromosomes 5D and 7B also showed pleiotropic effects for CTV and DM in non-stressed and heat stressed conditions. The outcomes of the current experiment are timely in relation to developing efficient molecular markers and determining the function of related genes. The significantly associated SNP markers and genomic regions recognized would be useful for marker-assisted selection for heat tolerant wheat breeding scheme.

## Supporting information

S1 File (DOC)
